RETRACTED

# The quality of life among Sudanese patients with epilepsy, Khartoum, Sudan

**DOI:** 10.1002/brb3.2487

**Published:** 2022-01-18

**Authors:** Etedal A. Ahmed Ibrahim, Lina Hussain Mustafa Ali, Khabab Abbasher Hussien Mohamed Ahmed, Mohammed Eltahier Abdalla Omer, Ibrahim M. Mahgoub, Mazin Salah‐Eldien Hassan Haroun, Moez Mohammed Ibrahim Bashir

**Affiliations:** ^1^ Faculty of Medicine Al Neelain University Khartoum Sudan; ^2^ The National Centre for Neurological Science Khartoum Sudan; ^3^ Faculty of Medicine University of Khartoum Khartoum Sudan; ^4^ Department of Internal Medicine Faculty of Medicine and Health Sciences Gadarif University Gadarif Sudan

**Keywords:** epilepsy, quality of life, Sudan

## Abstract

**Introduction:**

This is the first study done in the National Center for Neurological Sciences, Khartoum State, to assess the quality of life among more than 100 Sudanese epileptic patients, in the period from September to December 2020.

**Methodology:**

This is a descriptive cross‐sectional study; data were collected using an interview‐based semi‐structured structured questionnaire and this questionnaire was modified from the SF‐36 model.

**Results:**

Most of the patients were from urban areas and origin (60.2%), most of which were housewives; the majority of the patients were single and from low socioeconomic status, history of the disease was less than 3 years for most of the cases covered in this study, most of the cases were classified as generalized tonic clonic epilepsy, and normal EEG findings and normal MRI brain were found in 75.7% and 78.6%, respectively. Most patients mentioned that they experienced no attacks during the last month. Regarding mental health, 47.6% experienced symptoms of depression, and 75.7% had memory problems. In terms of physical health, 51.5% felt energetic all of the time, 9.7% experienced remarkable sleep disturbance, most of the patients are not driving nor have established hobbies during leisure time. 63.1% of the participants do not have health problems; 32% mentioned that they would feel stigmatized if an attack takes place in public. Commonest medication prescribed was carbamazepine, out of which 73.8% are fully compliant with their medication. 95.1% are not worried about long term use of medication.

**Conclusion:**

Lower levels of education and manual labor are associated with poor quality of life. Epilepsy has an adverse impact on social life. There is a global decrease in cognitive function, and most of the patients are not worried about the side effects and duration of the medication usage.

## Abstract 2

1 This is the first study done in the National Center for Neurological Sciences, Khartoum State, to assess the quality of life among more than 100 Sudanese epileptic patients.

2 Quality of life in patients with brain disorders is less in comparison with individuals from the general population; it is negatively comparable and/or worse in epilepsy patients than that in patients with other chronic conditions.

3 In this national study, we found that lower levels of education and manual labor are associated with poor quality of life, epilepsy has an adverse impact on social life, there is a global decrease in cognitive function, and most of the patients are not worried about the side effects and duration of the medication usage.

RETRACTED

## 1 BACKGROUND

Epilepsy is a group of neurological disorders characterized by recurrent seizures that can range from short, barely detectable episodes to prolonged episodes of intense tremors caused by abnormal electrical activity in the brain. These episodes can lead to physical injury, direct fractures, or accidents. In epilepsy, seizures tend to recur and have no immediate underlying cause. Isolated seizures caused by a specific cause, such as poisoning, and these are not considered epilepsy.

Seizures can occur in the cerebral cortex or subcortical structures. Using a detailed history, EEG results, and additional information, the doctor can usually classify the seizure and the epileptic type, followed by developing an appropriate treatment plan and adequate diagnostic assessment.

Subtypes of generalized seizures are categorized as: absence, generalized tonic clonic (GTC), atonic, and myoclonic. Absence seizures (petit mal) take the characteristic presentation of staring or daydreaming with a lack of response to external stimuli, typically with head cernuous or eye blinking. GTC seizures (grand mal) involve impairment of consciousness with bilateral radially symmetrical convulsive movements (stiffening followed by jerking) of all limbs. Myoclonic seizures are sudden, transient (“lightning‐fast”) movements however not related to any disturbance of consciousness.

(Secondary generalized epilepsy) Bilateral partial tonic‐clonic seizure is a type of seizure that begins in one region of the brain and then spreads to both sides of the brain as a tonic‐clonic seizure, characterized by short, involuntary muscle contractions that may affect one or more groups of muscle; therefore, myoclonic seizures can become generalized or focal. Atonic seizures effect as in loss of body tone, often leading to drooping of the head or whole body drooping (Berg & Millichap, 2013; Berg et al., 2010; Muro & Connolly, 2014). The clinical manifestations of a focal seizure depend on the area of the cerebral cortex affected. For example, a focal seizure arising from the prepsychotic cycle is manifested by asexual or tonic rhythmic locomotor activity, the occipital lobe with visual phenomena, and the posterior ileum with sensory symptoms such as paresthesia.

RETRACTED

The seizure is assessed as dyscognitive (formerly known as advanced partial) when consciousness is impaired throughout a raptus, means the patient is unable to retort remarkably to verbal stimuli; seizures arising from the lobe are often dyscognitive. An aura precedes a focal dyscognitive or grand mal seizure by seconds or minutes and is most frequently full‐fledged in patients with temporal lobe epilepsy. An aura could be a focal seizure whereby a patient retains awareness and describes sensory, motor, autonomic, or psychic symptoms.

The WHO has outlined QOL as “an individual” perception of their position in life within the context of the known culture and worth systems within which they live and in respect to their goals, expectations, standards, and concerns (Group, 1996).

Quality of life in patients with brain disorders is less in comparison with individuals from the general population; it is negatively comparable and/or worse in epilepsy patients than that in patients with other chronic conditions; in cases of well controlled epilepsy, the QOL is remarkably better as a result of their apprehension to the general matters and risks of the disease. Frequency of seizures appears to be one of the highly relevant determinants of poor quality‐of‐life (QOL) scores; quality of life becomes additionally worse and extremely unhealthy with the presence of depression; there are no contradicting results obtainable regarding the impact of drug treatment. Role activities, emotional perception, and noesis are the foremost investigated domains of quality of life in brain disorder research. Currently, the standard of life and psychosocial functioning in individuals with epilepsy are being investigated in several studies with continuously expanding manners (Berto, 2002).

Epilepsy may be a common chronic neurological disease that conveys a remarkable impact on people's lives including, but not limited to the social, physical, and emotional terms (Baker et al., 1997; Forsgren et al., 2005; Strine et al., 2005; Van Andel et al., 2009).

The recurrence of seizures is unpredictable and may cause mental health effects; it may as well build a perception of danger in patients, in addition to increased episodes of depression particularly when seizures take place in a public area (Ronen et al., 2003).

Stigma is a huge drawback to epileptic patients, which inevitably leads to the patient's life being restricted socially, increasing the work difficulties, and leading to poor QOL (Jacoby, 2008; Olsson & Campenhausen, 1993; Raty & Wilde Larsson, 2007; Smeets et al., 2007).

RETRACTED

In previous studies, QOL was assessed using many instruments in several community sectors (e.g., patients, workers, general population). SF‐36 questionnaire is one of these instruments, a generic instrument translated and valid in Islamic Republic of Iran by Montazeri (Montazeri et al., 2005).

Data concerning QOL in a highly detailed manner is incredibly necessary to assist healthcare professionals and medical employees generally in delivering higher quality of services to patients through implementation and intervention (Baker et al., 2005; Guekht et al., 2007; Mrabet et al., 2004; Phabphal et al., 2009; Shakir & Al‐Asadi, 2012; Stavem et al., 2000).

## 2 OBJECTIVES

### 2.1 General objective

General objective is to assess the mental health and the quality of life among epileptic patients aged 18–60 years and to correlate it with the control of the disease.

### 2.2 Specific objectives

- To assess mental health among epileptic patients.
- To assess physical health among epileptic patients.
- To assess the compliance of medication among epileptic patients.
- To assess the life restrictions regarding daily activities, occupation, social status, and hobbies, among epileptic patients.

## 3 METHODOLOGY

This is a descriptive cross‐sectional hospital‐based study. It was conducted in the tertiary hospital of neurological sciences in the National Neurological Center Clinic, considered one of the main reference teaching hospitals in Sudan. In this center there are several facilities including the main laboratory which includes stem cell laboratory and general laboratory, an X‐ray department, blood bank, pharmacy, physiotherapy department, and ICU. The NCNS center has two wards, medical and surgical. With a 110 beds capacity, with 24 of them in the medical ward. The medical ward receives almost 650 patients annually. There are four outpatient clinics. These clinics receive referred patients from all over Sudan which are estimated to be about 3000 patients annually. The study was conducted during the period from September to December 2020. The sample size was 103 patients. The study population included all patients who were diagnosed with epilepsy and admitted to the hospital, within the study period, and fulfilled the following criteria:

### 3.1 Inclusion criteria

- Adult patients aged from 18 to 60 years.
- Patients diagnosed with epilepsy and on anti‐seizures medications.
- Patients visiting neurological clinics in the National Centre for Neurological science within the study time period.
- Patients who accepted to participate in the study.
- Patients in a stable clinical condition at the time of assessment.

RETRACTED

### 3.2 Exclusion criteria

- Individuals not fulfilling the inclusion criteria.
- Non‐Sudanese patients.
- Patients who are known to have secondary epilepsy due to structural disease.

### 3.3 Data collection

Data were collected using a semi‐structured interview‐based questionnaire; section A: including age, gender, residence, education, occupation, marital status, socioeconomic status, family history. Section B included quality of life (score 10/10), duration of the disease, type of epilepsy, EEG changes, MRI brain findings, duration of medication, attacks in last month, type of medication in use, single or multiple medication, compliant with medication or not, side effects experienced, worry levels about using the medication. Section C: including mental and physical health (nervousness, memory status, depression, concentration, energy levels, sleep disturbances). Section D: social life (leisure time, driving, work/occupation, social activities), “Do you worry about hurting yourself during a seizure?”, “How worried are you about embarrassment or other social problems resulting from having a seizure in public?”, “How good or bad do you think your health is?” (measured in score 100/100). This questionnaire was modified from SF‐36 model.

### 3.4 Data analysis

The data were analyzed by a computerized program, statistical package for social sciences (SPSS) and results are presented in tables and figures.

### 3.5 Ethical approval

A written ethical clearance and approval for conducting this research was obtained from The National Centre for Neurological Science's ethical committee. Both verbal and written consents were taken from all participants before conducting the study. All subjects were informed that all the collected data were used for the research purpose only.

## 4 RESULTS

### 4.1 Demographic characteristics

The study age groups ranged from 18 to 60 years: 61.2% of them were in the age group (18 to 30 years) (Table 1). The mean age was 1.73 +/− 1.05 years; the second age group was from 31 to 40 and represented 16.5%; 41–50 years, 10.7%; and last group 51 to 60 years, 11.7%. Male to female ratio was 1:1.1 (46.6% male, 53.4% female). Most of the patients originated from urban areas (60.2%) followed by rural areas (39.8%). 41.7% of patients only reached primary levels of education in school, 11.7% were not educated. The patients educated at university levels represented 20.4% and secondary school 26.2%. Housewives were the most cases collected in this study (37.9%); labors represented 26.2%. Only two patients were employees (1.9%). Other occupations such as student, teacher, and others represented 34%. Most of the participants enrolled were single, 57.3%; 37.9% were married, three cases were divorced, and 1.9% widows. Most of the cases have low income (89.3%), while 10.7% had middle income. Family history of the same condition was relevant in 18.4%, and finally 81.6% had no family history of epilepsy.

RETRACTED

**TABLE 1:** Demographic data among 103 Sudanese epileptic patients

Variable				
Age	18–30 years (61.2%) *n* = 63	31–40 years (16.5%) *n* = 17	41–50 years (10.7%) *n* = 11	51–60 years (11.7%) *n *= 12
Gender	Male 46.6% *n *= 48	Female 53.4% *n* = 55		
Residence	Urban 60.2% *n* = 62	Rural 39.8% *n* = 41		
Education	Illiterate 11.7% *n* = 12	Primary 41.7% *n* = 43	Secondary 26.2% *n* = 27	University or above 20.4% *n* = 21
Occupation	House wife 37.9% *n* = 39	Laborer 26.2% *n* = 27	Employee 1.9% *n* = 2	Others 34% *n *= 35
Marriage	Single 57.3% *n* = 59	Married 37.9% *n* = 39	Divorced 2.9% *n* = 3	Widow 1.9% *n* = 2
Socioeconomic	Low 89.3% *n* = 92	Middle 10.7% *n* = 11		
FH of epilepsy	Positive 18.4% *n* = 19	Negative 80.4% *n* = 84		

### 4.2 Quality of life

The self‐assessment of patients about their lives was good 31.1% (in score language 10/10) (Table 2). Only one case considered himself 1 out of 10, 2.9% in 2, 6.8% in 4, 31.1% in 6, 27.2% in 8. The mean of the score to assess the quality life was 7.4 +/− 2.2.

**TABLE 2:** Quality of life among 103 Sudanese epileptic patients

	Frequency	Percent
1	1	1.0
2	3	2.9
4	7	6.8
6	32	31.1
8	28	27.2
10	32	31.1
Total	103	100.0

20.4% mentioned being diagnosed more than 15 years ago, while most of the cases were diagnosed less than 3 years ago (28.2%) and only 5.8% in duration from 8 to 10 years, 5 to 8 years 13.6%, and 13.6% in duration 10 to 15 years (Table 3).

**TABLE 3:** For how long have been diagnosed among 103 Sudanese epileptic patients

	Frequency	Percent
1–3 years	29	28.2
3–5	18	17.5
5–8	14	13.6
8–10	6	5.8
10–15	14	13.6
More than 15	22	20.4
Total	103	100.0

The most diagnosed type of epilepsy was generalized tonic clonic seizures which included 63.1% of cases, followed by simple partial and focal to bilateral each represented 7.8%, and myoclonic represented 1%, temporal epilepsy was 5.8%, complex partial (4.9%), absence (4.9%), and atonic 2.9% (Table 4).

**TABLE 4:** Type of epilepsy among 103 Sudanese epileptic patients

	Frequency	Percent
Generalized tonic clonic	65	63.1
Simple partial (focal)	8	7.8
Complex partial (focal)	5	4.9
Absence	5	4.9
Myoclonic	1	1.0
Tonic	2	1.9
Focal to bilateral	8	7.8
Temporal	6	5.8
Atonic	3	2.9
Total	103	100.0

Only 24.3% of the cases were associated with EEG abnormalities; 75.7% showed normal findings. Generalized tonic clonic patients who had EEG changes were in the form of generalized epileptiform discharge, temporal epilepsy associated with temporal epileptiform discharge, focal to bilateral frontotemporal epileptiform discharge (Table 5).

RETRACTED

**TABLE 5:** EEG changes among 103 Sudanese epileptic patients

	Frequency	Percent
Yes	25	24.3
No	78	75.7
Total	103	100.0

MRI brain detected abnormalities in 21.4% of cases; 78.6% were normal. Findings of MRI were gliotic changes, infarctions, and mesial temporal sclerosis, mostly noticed in generalized tonic clonic and temporal epilepsy (Table 6).

**TABLE 6:** MRI changes among 103 Sudanese epileptic patients

	Frequency	Percent
Normal	81	78.6
Abnormal	22	21.4
Total	103	100.0

41.7% of participants’ duration of treatment was from 1 to 3 years, 16.5% of cases from 3 to 5 years; patients who continued on treatment more than 15 years represented 13.6%, and 11.7% from 5 to 8 years, 3.9% 8 to 10 years, and 12.6% from 10 to 15 years (Table 7).

**TABLE 7:** How long he/she has been on antiepileptic among 103 Sudanese epileptic patients

	Frequency	Percent
1–3	43	41.7
3–5	17	16.5
5–8	12	11.7
8–10	4	3.9
10–15	13	12.6
More than 15	14	13.6
Total	103	100.0

Most of the patients mentioned having no attacks of seizure during the last month (47.6%), 36.6% associated with 1 to 2 attacks in the last month, and 15.5% associated with three to five attacks in the last month (Table 8).

**TABLE 8:** Attacks in the last month among 103 Sudanese epileptic patients

	Frequency	Percent
No attacks	49	47.6
1–2	38	36.9
3–5	16	15.5
Total	103	100.0

16.5% mentioned that they developed a more nervous personality, while 56.3% mentioned having no change in personality. One case mentioned feeling depressed all of the time. 47.6% felt depressed sometimes and 40.8% felt no kind of depression. 75.7% mentioned having memory problems and deficits. 55.4% of patients recorded having difficulty in concentrating during reading. 45.6% could do any task without problems, while 54.4% associated with problem completing and concentrating on tasks. 51.5% of the enrolled patients recorded feeling energetic all of the time and 1% mentioned always feeling tired with a lack of energy. About 9.7% mentioned having remarkable sleep disturbances (Table 9).

**TABLE 9:** Mental and physical health among 103 Sudanese epileptic patients table

	Nervous patients	Depression	Memory problem	Reading trouble	Concentrating trouble	Feel energetic	Feel tired	Sleep disturbance
All of the time	0% *n* = 0	1% *n* = 1	2.9% *n* = 3	21.4% *n* = 22	1.9% *n* = 2	51.5% *n* = 53	1% *n* = 1	0% *n* = 0
Most of the time	16.5% *n* = 17	10.7% *n* = 11	35% *n* = 36	34% *n* = 35	22.3% *n* = 23	31.1% *n* = 32	12.6% *n* = 13	9.7% *n* = 10
A little of the time	27.2% *n *= 28	47.6% *n *= 49	37.9% *n* = 39	17.5% *n *= 18	30.1% *n *= 31	17.5% *n *= 18	38.8% *n *= 40	20.4% *n* = 21
None of the time	56.3% *n *= 58	40.8% *n* = 42	24.3% *n* = 25	27.2% *n* = 28	45.6% *n* = 47	0% *n* = 0	47.6% *n* = 49	69.9% *n* = 72

Most of the cases have no leisure time (42.7%). 90.3% of patients do not drive. Work limitations were significant in 46.6% of the enrolled individuals. 9.7% of the individuals mentioned experiencing work limitations most of the time and 35% do not have any work limitations at all. 63.1% of the cases recorded no social limitations. Furthermore, 63.1% have no health problem preventing them from participating in social activities (Table 10).

RETRACTED

**TABLE 10:** Social life of epileptic patients among 103 Sudanese epileptic patients

	Leisure time	Driving	Work limitation	Social limitation	Social activities
A lot	4.9% *n* = 5	4.9% *n* = 5	46.6% *n *= 48	1.9% *n *= 2	1.9% *n *= 2
Most of time	7.8% *n* = 8	0% *n *= 0	9.7% *n* = 10	15.5% *n* = 16	15.5% *n* = 16
Only a little	8.7% *n* = 9	1% *n *= 1	8.7% *n *= 9	19.4% *n* = 20	19.4% *n* = 20
Not at all	35.9% *n* = 37	3.9% *n* = 4	35% *n* = 36	63.1% *n* = 65	63.1% *n* = 65
None	42.7% *n *= 44	90.3% *n* = 93	———–	———–	———–

31.1% were worried about themselves being hurt during seizures (Table 11).

**TABLE 11:** Do you worry about hurting yourself during a seizure among 103 Sudanese epileptic patients

	Frequency	Percent
Worry a lot	3	2.9
Occasionally worry	29	28.2
Do not worry at all	71	68.0
Total	103	100.0

32% of the participants feel embarrassed if the attack of the seizure happens in public (Table 12).

**TABLE 12:** How worried are you about embarrassment or other social problem resulting from having a seizure in public among 103 Sudanese epileptic patients

	Frequency	Percent
Worry a lot	12	11.7
Occasionally worry	21	20.4
Do not worry at all	70	68.0
Total	103	100.0

If physical health was allocated in scores ranging from zero to 100, most of the patients put themselves in 79 +/− 14 (Table 13).

**TABLE 13:** How good or bad do you think your health is among 103 Sudanese epileptic patients

	Frequency	Percent
50	5	4.9
60	11	10.7
70	23	22.3
80	28	27.2
90	16	15.5
100	20	19.4
Total	103	100.0

The commonest medication prescribed was carbamazepine and 64.1% of patients were using it, followed by sodium valproate, 41.7% were using it. No one used phenytoin. 7.8% were using lamotrigine, 12.6% were on levetiracetam, tobriamate was used by 1%, and 27.2% of the patients were on multiple medications.

73.8% were compliant with medications all of the time, 6.8% a little of the time, and 19.4% most of the time.

25.2% recorded experiencing side effect from medications, and most side effects were nausea (9.7%), dizziness (5.8%), drowsiness (6.8%), and others represented 2.9%; finally 74.8% of patients experienced no side effects.

95.1% of patients were not worried about the long‐term use of medication, with the remaining percentage of participants remarkably worried.

RETRACTED

## 5 DISCUSSION

This is the first study done in the National Center for Neurological Science to assess the overall quality of life of Sudanese patients with epilepsy and to assess the struggles that affect their quality of life.

In our study, the mean age was 22 years, in comparison with a study done in rural area of Chaco, which showed a similar mean age of 24.2 years (Nicoletti et al., 2018).

In our study, the gender distribution was 46.6% male and 53.4% female. Female distribution was slightly higher in comparison with a study published from Europe, which classified the incidence of epilepsy according to gender, and accordingly there was no difference between male and female gender (1:1) (Christensen et al., 2005). In our study, 41.7% of the patients graduated from primary school, 11.7% were not educated, patients educated from universities represent about 20.4%, and secondary school 26.2%. According to this set of data, we have considerably higher levels of education than in Ethiopia. Educational status in Ethiopia among epileptic patients was (27.6%) secondary school, (26.8%) primary school, and 18.1% completed university or higher studies (Abadiga et al., 2019).

Moreover, a study done in a high‐income area associated with higher levels of education, Saudi Arabia, showed the educational level in epileptic patients to be 68.38% among males and 63.07% among females, and this subset of the sample received a Diploma or a bachelor's degree. This is highly associated with more compliance to treatment and awareness regarding their illness and in turn helps them to avoid risk factors that may exaggerate and exacerbate the seizure attacks, which eventually leads to better quality of life (Alshahrani et al., 2019). In Sweden, the most dominant occupation in epileptic patients was manual work (82.2%) and then professionals to a lesser extent (17.8%). Arguably, the manual worker groups were at higher risk for occupational hazards than professional jobs; this in turn affects the health of patients in adverse ways (Li et al., 2008). In our study, housewives represented the highest proportion among the samples collected (37.9 %); manual workers represented 26.2 %; patients with professional jobs represented 35.9%. This indicates higher safety indices as professional job occupants are at lesser risks of acquiring or experiencing attacks, as well as decreased exposure to occupational hazards when compared to manual workers, which does not go in line with a similar study conducted on Swedish epileptic patients, where manual workers represented a larger proportion of the studied sample. The impact of epilepsy is arguably negative on the income and occupation of the patients. A study conducted in Sudan shed light on results that stated that 17% of the patients of the studied sample were unemployed or had their job terminated as a result of epilepsy, and these definitely led to financial difficulties which compromised their access to anti‐seizures medications (Sokrab et al., 2012).

RETRACTED

In our study, most of the enrolled patients were single (57.3%); 37.9% were married, 2.9% were divorced, and 1.9% were widows. The high levels of single marital status clearly reflects the social stigma associated with epilepsy, as a vast majority of the population believes this disease is familial and can be inherited. In a similar research study conducted in China where patients were generally observed for a period of 5 years, with results showing that 46.4% were single and 9.1% were divorced, it was evident that epilepsy in China had more prominent effects on patients’ social life than in Sudan; therefore, both our study and the study conducted in China reflected a remarkably unstable social life (Wada et al., 2004).

In our study, most of the cases have a low‐income level (89.3%); 10.7% with middle income. In comparison with a study done in Sweden which revealed that the low‐income group represented 48.5% of the sample, middle income represented 31.1% and high income 20.3%. Regardless of the fact that the Swedish population has higher income levels when compared to Sudan, it is evident that it has a higher percentage of manual workers, thus exposing the patients to more occupational hazards in Swedish patients (Li et al., 2008). In this study, the family history of the same condition was prevalent in (18.4%). In another study conducted by Ottman et al., there is a strong correlation between epilepsy and positive parents with epilepsy, which reached up to 32% (Ottman et al., 2011).

In our study, the self‐assessment/evaluation of patients regarding their lives was good (31.1%) (in a scored manner of 10/10). In Ethiopia, more than half of the enrolled patients mentioned leading a good quality of life (54.8%) which is significantly higher than the results provided by our study. Although Sudanese educational levels are generally higher, the impacts are still apparent. The lower self‐assessment/evaluation among the Sudanese patients may be attributed to the overall satisfaction of the patients with the healthcare system and the QOL factors related to it, in addition to the general awareness of the patients (Abadiga et al., 2019; Muche et al., 2020).

RETRACTED

In our study, the generalized tonic clonic seizure represented 63.1%, partial represented 7.8%, and focal to bilateral represented 7.8% of the patients. While in another study done by Keränen et al., distribution of epilepsy according to type was 44% generalized tonic clonic seizure, 23% had partial complex seizure, 7.5% simple partial seizure, and 25.5% with focal to bilateral seizures (Keränen et al., 1988).

In our study, only 24.3% were associated with EEG abnormality changes; 75.7% showed normal findings. This was not in line with another study where 75% showed EEG changes (Britton et al., 2016). In this study, MRI brain detected abnormalities in 21.4%, and 78.6% were normal. While another study done by Cendes et al. showed the positive finding in MRI of epileptic patients was 40% (Cendes et al., 2016).

In our study, most of the patients that mentioned having no attacks of seizures during the last month represented 47.6%; 36.6% mentioned experiencing one to two attacks during the last month and 15.5% were associated with three to five attacks in the last month. In a similar study conducted in Ethiopia, it was reported that patients that experienced one attack per month represented 14.2%, two attacks in 13.4%, three attacks per month in 7.6%, and about 60% completely free from attacks. Generally speaking, Sudan has higher educational levels compared to Ethiopia, but in Ethiopia, there is a better quality of life, and this may be associated with the frequency of attacks experienced as well as levels of controlling of disease (Tigistu et al., 2018).

In our study, 16.5% of the enrolled patients mentioned that they developed a nervous personality as a result of the epilepsy, while 56.3% mentioned having no personality changes. A study done by Gnanavel et al. showed high levels of depression among epileptic patients which reached up to 55% (Gnanavel, 2017). This goes in line with the results in our study, where one case reported feeling depressed all of the time, 47.6% reported experiencing depression “sometimes”, and 40.8% felt no depression at all.

In our study, 75.7% mentioned experiencing problems with memory, 55.4% of patients reported difficulties in concentrating on reading, 45.6% can complete various fundamental tasks without problems, and 54.4% reported having problems completing and concentrating on tasks. When comparing these results to a study conducted by Hermann et al., there is a global decrease and impairment of the cognitive function in 47% of the cases (Hermann et al., 2007).

RETRACTED

In our study, 51.5% reported feeling energetic all of the time and 1% reported feeling tired almost all of the time; about 9.7% mentioned having sleeping disturbances all of the time. In a similar research conducted by Bjrholt et al., the results showed an overall lower level of physical activity when compared to enrolled patients in our study (Bjrholt et al., 1990).

Work limitation was experienced by 46.6% a lot of the time, while 35% had no limitation in work. In another study conducted, the work limitation was found to be 42% (Volpato et al., 2017).

In our study, 63.1% has no social limitation and 63.1% has no health problem to prevent social activities; 31.1% are worried about themselves being hurt during seizures; 32% reported being embarrassed if the seizure attacks take place in public. When comparing this study with a previous study done in Sudan, 58% had no social activities, 15% feel stigmatized with epilepsy, and this study mentioned injuries during seizures were evident in up to 52% (Sokrab et al., 2012). When allocating the physical health in scores from a total of 100, most of the patients put themselves in 79 +/− 14, similar to the results from a study conducted by Volpato et al. (2017).

In our study, the commonest medication prescribed was carbamazepine and 64.1% of the patients were using it, followed by Na valproate and about (41.7 %) were using it; no one used phenytoin. 7.8% were using lamotrigine. Levetiracetam was used by 12.6%, tobriamate by 1%, and 27.2% of the patients were on multiple medications. In India, prescription of monotherapy and polytherapy with two and greater than or equal to three AEDs in 37.9%, 34.9%, and 27.2% patients, respectively was reported (Joshi et al., 2017). In Ethiopia, 63.41% of the participants were taking two antiepileptic medications and associated with more side effects (Hasiso & Desse, 2016). In Ethiopia, the most frequently prescribed medications used were phenobarbital (67%) and phenytoin (33.3%) (Nasir et al., 2020). In our study, about 73.8% were compliant with the medication all of the time, 6.8% were compliant in a little proportion of the time, and 19.4% were compliant most of the time. In Ethiopia, 32% of the patients in their study were adherent to treatment, and the most reported causes for non‐adherence were forgetfulness (75.4%) and running out of pills (10.8%). In our study, we have a higher percentage of compliance, and this may be due to higher percentage of the monotherapy than polytherapy in our patients (Hasiso & Desse, 2016).

In our study, 25.2% reported experiencing significant side effects from the medications, and most side effects reported were nausea (9.7%), dizziness (5.8%), drowsiness (6.8%), and others represent 2.9%. The remaining 74.8% reported experiencing no side effects. When these results are compared with a previous study done in Sudan, it showed the same side effects of medications where 26% experienced one or more side effects (Sokrab et al., 2012).

RETRACTED

Moreover, another study in India showed different results in terms of the experienced side effects: nausea (5.3%), dizziness (5.6%), drowsiness (40.1%), memory problems (30.3%), headache (28%), tiredness (34%) (Joshi et al., 2017). In our study, 95.1% of the patients were not worried about the long‐term usage of medication, 4.9% were worried. When comparing these results with a study done in Ethiopia, the patients were more worried about using the anti‐seizure medications than in our study; about 67.4% were worried about the long‐term usage of the medication (Nasir et al., 2020).

## 6 CONCLUSION

Most of the epileptic patients are housewives. Lower levels of education and manual labor are both associated with poor quality of life, especially manual laborers who are exposed to higher occupational hazards than professional job occupants, and this eventually has negative impacts on income. Epilepsy has negative effects and impacts on social life. The most common type of epilepsy in our study is generalized tonic clonic seizure. The majority of epileptic patients have normal EEG. Depression rates in our study are similar to international studies. In our study, there is global decrease in cognitive functions, which is similar worldwide. The compliance with medication in our study was good. Most of patients in our study did not mention worrying about medications’ side effects and long‐term usage.

## FUNDING INFORMATION

The authors received no specific funding for this work.

## CONFLICT OF INTEREST

The authors have no conflict of interest to declare.

## AUTHOR CONTRIBUTIONS

All authors read and approved the final manuscript.

### PEER REVIEW

The peer review history for this article is available at https://publons.com/publon/10.1002/brb3.2487

## Data Availability

The datasets used and∖or analyzed during the current study are available from corresponding author on reasonable request.
